This article has been retracted.

# Clinical Significance of EZH2 in Acute Myeloid Leukemia

**DOI:** 10.1155/2022/8741989

**Published:** 2022-08-23

**Authors:** Weiyun Jiao, Yuanyuan Liu, Yangyi Bao

**Affiliations:** Hematology Department, Hefei First People's Hospital, Hefei 23000, China

## Abstract

In this paper, we have focused on the investigation of the expression level of the enhancer of zeste homolog 2 (EZH2) gene in bone marrow mononuclear cells of acute myeloid leukemia (AML) patients and analyze the relationship between EZH2 gene expression and EMI. The expression of EZH2mRNA in bone marrow mononuclear cells of 26 patients with incipient AML was detected by qRT-PCR, and the relationship between EZH2mRNA expression and clinical characteristics was analyzed. EZH2 mRNA expression was increased in 26 AML patients. EZH2 gene expression in male patients was significantly higher than that in female patients. The expression of EZH2 in the group with extramedullary infiltration (EMI) was significantly higher than that in the group without EMI. The patients were divided into different groups according to the chromosomal karyotype and prognosis. Statistical analysis showed that the expression level of the medium-risk group was significantly higher than that of the low-risk group, while there was no statistical difference in other groups (*P* > 0.05). The expression of EZH2 gene in AML patients was closely related to EMI, and the expression of EZH2 in AML cells was closely related to cell migration ability. EZH2 is expected to be one of the indicators of disease recurrence.

## 1. Introduction

Acute myeloid leukemia (AML) is a malignant tumor of hematopoietic stem and progenitor cells. The malignant proliferation of leukemia cells gradually replaces normal hematopoiesis in the body and invades extramedullary tissues and organs, resulting in anemia, bleeding, infection and organ enlargement, and ultimately death. In recent years, with the rapid economic development and increasingly serious environmental pollution, the annual incidence of leukemia is on the rise [1]. New epidemiological survey data show [2] that the mortality rate of leukemia in my country is as high as 4.28/10. It ranks eighth in malignant tumors.

AML is the most common type of adult leukemia. At present, with the emergence of new chemotherapy drugs and the continuous improvement and innovation of chemotherapy regimen, the remission rate of leukemia treatment has been significantly improved. 50–85% of AML patients can obtain complete response (CR) after standard regimen induction therapy [3]. The use of high-intensity consolidation chemotherapy and hematopoietic stem cell transplantation has made the long-term survival rates to improve, but most patients will relapse after reaching CR and develop drug resistance to chemotherapy drugs or even progress to refractory leukemia and eventually death.

Considering that EZH2 plays an important role in malignant tumors and is closely related to tumor invasion and metastasis and poor prognosis, there are few studies on the overexpression of EZH2 in leukemia and its clinical significance. Therefore, in this study, the expression level of EZH2 gene in bone marrow mononuclear cells of AML patients was detected by qRT-PCR, and the relationship between its expression and clinical characteristics, treatment response, and prognosis were analyzed, providing a new indicator for the diagnosis, treatment, and prognosis evaluation of leukemia.

The enhancer of zeste homolog 2 (EZH2) plays the role of a proto-oncogene in malignant solid tumors, while hematological tumors have two states of gain and loss of function, which play a role in promoting or inhibiting cancer. EZH2 was found to be involved in the occurrence and development of AML. Momparler et al. [4] studied the function of EZH2 in AML in mice, and the results showed that in the artificially constructed AF9 positive AML model mice, the trimethylation level of H3K27 was significantly reduced in the EZH2-deficient group. The expression of genes related to cell growth and differentiation, such as Cdkn2a, increased significantly, suggesting that EZH2 inhibits the differentiation of leukemia stem cells in AML, thereby promoting the occurrence of leukemia. DZNep, as an EZH2 inhibitor, has a significant inhibitory effect on cell clonogenesis in both human and mouse AML cell lines and has an antileukemia effect in leukemia mouse models, accompanied by upregulated expression of tumor suppressor genes CDKN lA and FBX032 [5]. Domestic scholar Shenghao Wu found that EZH2 protein expression was significantly correlated with increased LDH, WBC, and shorter OS in bone marrow cells of AML patients. At the same time, EZH2 overexpression was accompanied by decreased miR-101 expression, suggesting that miRNA may have posttranscriptional regulation of EZH2 and promote the occurrence of leukemia [6].

In this paper, we have focused on the investigation of the expression level of the EZH2 gene in bone marrow mononuclear cells of AML patients and analyzed the relationship between EZH2 gene expression and EMI. The expression of EZH2mRNA in bone marrow mononuclear cells of 26 patients with incipient AML was detected by qRT-PCR, and the relationship between EZH2mRNA expression and clinical characteristics was analyzed. EZH2 mRNA expression was increased in 26 AML patients. EZH2 gene expression in male patients was significantly higher than that in female patients. The expression of EZH2 in the group with EMI was significantly higher than that in the group without EMI. The patients were divided into different groups according to the chromosomal karyotype and prognosis.

The remaining paper is organized as given in the following paragraph where a brief description of every section is provided.

In the subsequent section, a detailed discussion on the relationship between EZH2 gene expression and EMI is provided where it is clearly mentioned how data is collected. In Section 3, experimental results and observations are described in detail along with possible comparative evaluations which is followed by a brief discussion section. Finally, concluding remarks are provided at the end along with references.

## 2. Proposed Methodology

### 2.1. Participants

26 patients with newly treated AML in our hospital from June 2018 to June 2021 were retrospectively analyzed. All patients were confirmed by bone marrow morphological cytology, immunohistochemical staining, or flow cytometry immunotyping. All specimens were collected with the informed consent of the subjects or their families and approved by the hospital ethics committee.

### 2.2. Isolation of Bone Marrow Mononuclear Cells

Routine bone marrow puncture was performed to extract 3–5 mL of the patient's bone marrow fluid, heparin was anticoagulated, and bone marrow mononuclear cells were isolated by lymphocyte separation solution. After washing twice with PBS, 1 mL of Trizol was added, repeatedly beaten until no precipitation was found, and stored at −80°C for later use.

### 2.3. Total RNA Extraction

Total RNA was extracted according to Trizol instructions. After DEPC water was dissolved, the concentration and purity of RNA were determined by using a spectrophotometer. Only 2.0 >A260/A280 > 1.8 could be used for subsequent reverse transcription.

### 2.4. Reverse Transcriptional Reaction

Follow the instructions of TAKARA's Prime-Script reverse transcription kit. After fully mixing 1 *μ*g total RNA, 1 *μ*L Oligo(dT), and 18 *μ*L dNTPmix, the mixture was placed at 65°C for 5 min and then cooled quickly on ice. After adding 45 *μ* Prime-Script buffer, 1 *μ*L of the ribonuclease inhibitor, and finally, 1 *μ*L of enzyme mix reverse transcriptase (200 U/*μ*L) were added until the final volume was 20 *μ*. After being treated at 42°C for 1 h and 70°C for 10 min, cDNA was cooled on ice, and the first strand obtained was immediately PCR or stored in an 80°C refrigerator for future use.

### 2.5. Real-Time PCR

The SYBR Green fluorescence quantitative PCR(RT-PCR) kit was used for detection. The upstream primer of EZH2 was 5, -GACCCTGACCTCTGTCTTACTF-3, and the downstream primer was 5-GATgCTCCCAGGCAA AGATG-3. The upstream primer of internal reference GAPDH was 5″-TGAAGGTCGGAGTCAACGG-3, and the downstream primer was 5″ -CTGGAAGatGGTGATGGGATT-3. PCR amplification conditions were 95°C for 30 S, 95°C for 5 S, 60°C for 40 S, and 40 cycles. All reactions are set with 3 complex holes. The relative expression levels of target genes in the samples were expressed by the 2^−△△Ct^ method. The expression levels of the EZH2 gene were expressed as 2^−△△Ct^. The EZH2 mRNA of AML patients was multiplied by 10000, and 1 g of data was converted into a normal distribution and the Levene test for homogeneity of variance.

### 2.6. Statistical Analysis

SPSS23.0 statistical software was adopted to process the data. The measurement data were presented as ($\bar{x}\pm s$). The group design *t*-test was adopted for comparison, and the analysis of variance was adopted for comparison between multiple groups. The Dunnett's test was adopted for comparison with the control group. The counting data were presented in the number of cases, the percentage, *χ*^2^ test was adopted for comparison between the groups, and the bilateral test was employed for all statistical tests. Pearson correlation or Spearman rank correlation was used for correlation analysis. The Kaplan–Meier method was used for survival analysis. *P* < 0.05 was considered statistically significant.

## 3. Experimental Results

In this section, we are going to provide a detailed discussion on the effectiveness of the proposed scheme specifically with the supported experimental results which are collected through the implementation of the proposed procedure in the underlined environment.

### 3.1. Basic Characteristics of AML Patients

The 26 patients with AML included 18 bone marrow tissue samples and 8 extramedullary tissue samples (see Table 1 for the main clinical characteristics and treatment scheme). Through analysis and comparison of the clinical data of the two groups, it was found that the age, proportion of primary immature cells in the bone marrow, proportion of peripheral immature cells, WBC, LDH, disease status, FAB (M2/M4/M5/other) typing, and chromosome karyotype distribution of the two groups were basically the same, and there was no significant difference (*P* > 0.05), but there were significant differences in gender, initial induction scheme, and consolidation enhancement scheme between the two groups (*P* < 0.05), which provided a reference basis for analyzing the relationship between EZH2 protein expression and clinical characteristics after combining the data of the two groups.

*P* value is the comparison between the BM group and the EMI group; BM % and PB % were the proportion of bone marrow and peripheral blood protonaive cells, respectively. M2 in FAB included *L* patients with M1, 4 patients with undefined AML and 3 patients with granulocytic sarcoma. In the induction scheme, only *l* cases of HA and 2 cases of MA were incorporated into the DA and IA groups, respectively. Consolidation and reinforcement program: A represents induction program +<4 courses of MD/HD-Ara-c, B represents induction program +24 courses of MD/HD-Ara-C or Auto-HSCT, and C represents induction program + allo-HSCT. ^*∗*^ represents *P* < 0.05 and ^*∗∗*^ represents *P* < 0.01.

### 3.2. EZH2 mRNA Expression Level in Bone Marrow Cells of AML Patients

*T*-test results of two samples showed that the EZH2 gene expression level in AML patients was significantly higher than that in normal controls(*P* < 0.05). The expression level of EZH2 mRNA in bone marrow mononuclear cells of 42 AML patients was detected by RT-PCR. The expression level of EZI-12 mRNA in bone marrow cells of AML patients was 1.68 ± 0.73 (95%CI, 1.45–1.92). In the 10 normal controls, the rate was 0.87 ± 0.65(95%CI, 0.40∼1.34).

### 3.3. Expression and Clinical Characteristics of EZH2 mRNA in AML Patients

The expression of the EZH2 gene in the bone marrow of AML patients is closely related to the occurrence of EMI. In addition, the patients were divided into groups according to chromosome karyotype prognosis. The EZH2 gene expression level was 1.00 ± 0.05 in the low-risk group, 1.94 ± 0.60 in the medium-risk group, and 1.84 ± 0.64 in the high-risk group.The expression level of the EZH2 gene in bone marrow cells of AML patients was significantly correlated with males, proportion of juvenile cells in peripheral blood 30%, and WBC > 35 × 10^9^/*L* (*P* < 0.05) but not with the FAB type, age, proportion of juvenile cells in the bone marrow, LDH level, and complex karyotype (*P* > 0.05). Statistical analysis showed that there was no significant difference in the EZH2 expression level among the three groups (*P* > 0.05). However, the expression level of the EZH2 gene in the medium-risk group was significantly higher than that in the low-risk group (*P* < 0.05), suggesting that EZH2 may be one of the indicators for stratified diagnosis and prognosis assessment. According to whether patients were accompanied by EMI at the time of onset, patients were divided into the group accompanied by EMI and the group without EMI. The EZH2 gene expression level in the group accompanied by EMI was 2.04 ± 0.59, while that in the group without EMI was 1.29 ± 0.72. There was a significant difference Table 2 in the EZH2 gene expression level between the two groups (*P* < 0.05).

^*∗*^indicates a significant difference between the low-risk group and the medium-risk group; BM % represents the proportion of bone marrow naive cells, PB % represents the proportion of peripheral blood naive cells, and EMI represents extramedullary infiltration (EMI). ^*∗*^ represents *P* < 0.05 and ^*∗*^ represents *P* < 0.01.

## 4. Discussion

EMI is one of the malignant biological features of AML. The impact of EMI on prognosis is still a controversial issue, but most studies show that EMI is closely related to a lower CR rate, higher risk of relapse, and poor prognosis. Just like the invasion and metastasis of malignant tumor cells, the EMI process of leukemia cells is also a complex process involving multiple factors and completed by multiple steps [7]. Most scholars believe that the alteration of the bone marrow microenvironment and degradation of the extracellular matrix are leukemia cells. The mechanism of extramedullary infiltration of leukemia cells may involve abnormal expression of adhesion factors on the surface of leukemia cells. The ability of leukemia cell adhesion or migration is enhanced, and then escape from the adhesion of the bone marrow stroma and escape into the bone marrow stroma and peripheral blood, and then operate chemotactic movement and adhere to the vascular endothelium under the action of chemokines. It then promotes the secretion of cellular matrix metalloproteinases to degrade the extracellular matrix and migrate to extramedullary tissues to form infiltrating lesions [8].

A literature study has shown that EZH2 is overexpressed in a variety of malignant tumors, especially solid tumors, and its expression is related to patients' clinical stage, tumor malignancy, tumor invasion and metastasis, chemotherapy resistance, and poor prognosis [9].

In vitro culture of primary bone marrow cells from patients with cellular lymphoma found that the expression of EZH2 protein in proliferating cells was significantly higher than that in quiescent cell lines. In addition, it has been demonstrated that overexpressed EZH2 promotes lymphoma formation by regulating the immunoglobulin IgH rearrangement [10].

At present, epigenetic modification has become an important mechanism to regulate gene expression. It is a modification mode independent of DNA sequence changes, mainly including DNA methylation, histone covalent modification, and microRNA regulation. As a member of the PCG protein family, EZH2 is a catalytically active subunit of the PRC2 complex, which can induce trimethylation of histone H3K27 and then exert transcriptional inhibition on downstream target genes. Statistical analysis of the relationship between the expression of EZH2 and clinical features showed that EZH2 mRNA and protein expression were correlated with the proportion of peripheral blood naive cells, WBC, and associated EMI. In addition, EZH2 mRNA was also closely correlated with gender and karyotype prognosis stratigraphy, and the expression level of EZH2 mRNA in the medium-risk group was significantly higher than that in the low-risk group. Wu et al. [5] showed that the EZH2 mRNA expression level in bone marrow cells was not related to gender, WBC, and LDH, while EZH2 protein in bone marrow tissues was associated with WBC>. 1.50 × 109/*L* and increased LDH were significantly correlated, which was inconsistent with our results. In addition, this study believed that EZH2 mRNA and protein expression levels were inconsistent, which might be caused by the posttranscriptional regulation of EZH2 by Mir-101. Since our research group did not detect EZH2 mRNA and protein in the same specimen at the same time, and there are few studies in this area, it remains to be confirmed whether the mRNA and protein expression levels of EZH2 are consistent. Grubach et al. [11] and Tanaka al. [12] found that the expression level of the EZH2 gene in complex karyotype AML was significantly higher than that in normal AML patients. This study still has some shortcomings. Firstly, the quality of this study is limited due to the small sample size we included in the study. Secondly, this research is a single-center study, and our findings are subject to some degree of bias. Therefore, our results may differ from those of large-scale multicenter studies from other academic institutes. This research is still clinically significant, and further in-depth investigations will be carried out in the future.

## 5. Conclusion

The expression of the EZH2 gene in AML patients was closely related to EMI, and the expression of EZH2 in AML cells was closely related to cell migration ability. EZH2 is expected to be one of the indicators of disease recurrence. In this paper, we have focused on the investigation of the expression level of the EZH2 gene in bone marrow mononuclear cells of AML patients and analyzed the relationship between EZH2 gene expression and EMI. The expression of EZH2mRNA in bone marrow mononuclear cells of 26 patients with incipient AML was detected by qRT-PCR, and the relationship between EZH2mRNA expression and clinical characteristics was analyzed. EZH2 mRNA expression was increased in 26 AML patients. EZH2 gene expression in male patients was significantly higher than that in female patients. The expression of EZH2 in the group with EMI was significantly higher than that in the group without EMI. The patients were divided into different groups according to the chromosomal karyotype and prognosis.

In future, we are eager to extend the proposed study for the evaluation of the other metrics and different classes of patients in the smart healthcare domain.

## Figures and Tables

**Table 1:** Clinical characteristics and treatment of 26 patients with AML (median, range).

	*n*	BM (*n* = 18)	EMI (*n* = 8)	*X* ^2^/*Z*	*P*

Sex (M/F)	26	12/6	5/3	5.378	0.019^*∗*^
Age	26	34.2 (14.0–85)	32.8 (15–78.0)	−0.670	0.500
BM%	26	71.6 (24.8–93.6)	72.8 (23.7–92.4)	−0.500	0.615
PB%	26	45.8 (3.9–87.2)	46.7 (2.9–86.1)	−0.468	0.642
WBCx10^9^/L	26	12.5 (0.7–102.9)	12.2 (0.6–99.7)	−0.995	0.354
LDH	26	356 (140.2–924.7)	367.2 (143.5–938.1)	−0.399	0.692
Status (incipient/recurrent)	26	13/5	4/2	−0.388	0.685
FAB (M2/M4/M5/other)	26	5/2/10/1	5/0/1/2	7.602	0.056
Normal/complex karyotype	22	17/2	2/1	0.008	0.945
Prognostic stratification (low/medium/high)	25	5/12/1	1/4/2	2.747	0.256
Induce (DA/IA)	26	1/17	7/1	8.50	0.003^*∗∗*^
Consolidate (a/b/c)	20	10/1/4	4/2/0	8.299	0.015^*∗*^

**Table 2:** Relationship between the bone marrow EZH2 mRNA expression level and clinical features in 38 AML patients.

Clinical features	*N*	EZH2 mRNA	95CI%	*F*/*t*	*P*

Sex				2.718	0.010^*∗*^
Male	18	1.95 ± 0.65	1.65∼2.22		
Female	8	1.39 ± 0.67	1.04∼2.70		

Age				−0.496	0.627
	16	1.74 ± 0.72	1.42∼2.01		
	10	1.63 ± 0.68	1.23∼0.97		

FAB type				0.881	0.493
M1	2	1.55 ± 0.34	0.99∼2.11		
M2	6	1.72 ± 0.51	1.39∼2.01		
M3	4	1.92 ± 0.99	1.63∼2.63		
M4	8	1.49 ± 0.66	1.15∼1.84		

BM%				0.989	0.330
	10	1.55 ± 0.68	1.23∼1.91		
	16	1.79 ± 072	1.65∼2.22		

PB%				2.665	0.010^*∗*^
	8	1.33 ± 0.65	1.04∼1.75		
	18	1.95 ± 0.66	1.62∼2.24		

WBC				2.081	0.044^*∗*^
35	11	1.44 ± 0.75	1.05∼0.84		
35	15	1.93 ± 0.69	1.59∼2.05		

LDH				0.560	0.598
Normal	7	1.59 ± 0.98	0.58∼2.63		
Increase	19	1.78 ± 0.69	1.47∼2.06		

EMI				3.460	0.001^*∗∗*^
No	7	1.28 ± 0.71	0.93∼1.67		
Yes	8	2.05 ± 0.57	1.73∼2.30		

Karyotype				1.625	0.326
Normal	20	1.97 ± 0.61	1.69∼2.31		
Complex	6	1.54 ± 0.55	−5.39∼7.65		

Prognostic stratification				2.77	0.082
Low risk	4	1.00 ± 0.04	0.51∼1.46	−2.20	0.037^*∗*^a
Medium crisis	16	1.95 ± 0.58	1.72∼2.20		
High risk	6	1.84 ± 0.62	−0.56∼3.65		

## Data Availability

The datasets used and analyzed during the current study are available from the corresponding author upon reasonable request.
